# Geographical Inequality on Cataract Surgery Uptake in 200,000 Australians: Findings from the “45 and Up Study”

**DOI:** 10.1155/2022/9618912

**Published:** 2022-09-16

**Authors:** Guobei Xiao, Zhuoting Zhu, Xin Xiao, Zachary Tan, Ke Cao, Xianwen Shang, Karl D. Brown, Guofu Huang, Lei Zhang, Mingguang He

**Affiliations:** ^1^Department of Ophthalmology, The First Hospital of Nanchang, Nanchang, Jiangxi, China; ^2^Centre for Eye Research Australia, Royal Victorian Eye and Ear Hospital, East Melbourne, Victoria, Australia; ^3^State Key Laboratory of Ophthalmology, Zhongshan Ophthalmic Centre, Sun Yat-Sen University, Guangzhou, China; ^4^Centre for Optometry and Visual Science, People's Hospital of Guangxi Zhuang Autonomous Region, Nanning, China; ^5^School of Medicine, the University of Queensland, Brisbane, Queensland, Australia; ^6^Ophthalmology, Department of Surgery, University of Melbourne, Melbourne, Australia; ^7^Department of Epidemiology and Biostatistics, School of Public Health, Xi'an Jiaotong University Health Science Centre, Xi'an, China; ^8^Melbourne Sexual Health Centre, Alfred Health, Melbourne, Australia; ^9^Central Clinical School, Faculty of Medicine, Monash University, Melbourne, Australia; ^10^Department of Epidemiology and Biostatistics, College of Public Health, Zhengzhou University, Zhengzhou 450001, Henan, China

## Abstract

Using a geographical information system (GIS), we investigated the spatiotemporal evolution of a cataract surgery service and its association with socioeconomic factors and private insurance, based on 10-year real-world medical claim data in an Australian population. The data collected cover a decade (2007–2016) from the “45 and Up Study”. A total of 234,201 participants within the cataract surgery service were grouped into 88 Statistical Area Level 3 (SA3s) according to their residential postcodes in New South Wales Australia. We analyzed the spatiotemporal variations and geographical distribution inequality in cataract surgery incidence and its respect to socioeconomic status (SES) and private health insurance coverage by Spearman correlation analysis and Moran's I test. Then these variations were intuitive displayed by six-quartile maps and a local indicator of spatial association (LISA) maps based on GIS. The average cumulative age-gender-standardized of the incidence of cataract surgery (ICS) was 8.85% (95% CI, 5.33–15.6). Spatial variation was significant (univariate Moran's I = 0.45, *P* = 0.001) with incidence gradually decreasing from the coastal regions to the north-western inland regions, suggesting inequality in the cataract surgery service across the state of New South Wales. Notably, clustering of the low incidence areas had gradually disappeared over the decade, suggesting that the cataract surgery service has improved over time. Low scores on the “index of socioeconomic disadvantages” (IRSD) and high private health insurance coverage were significantly associated with a higher incidence of cataract surgery (bivariate Moran's I = −0.13 and 0.23, *P* < 0.01; Spearman correlation *r* = 0.25 and −0.25, *P* = 0.02), which is displayed on the map visually and obviously. Spatiotemporal variations in the incidence of cataract surgery are significant, but the low incidence area had gradually disappeared over time. High socioeconomic status and private insurance contribute to a higher incidence of cataract surgery in Australia.

## 1. Introduction

Cataract remains the major cause of visual impairment and blindness globally [1]. Vision loss due to cataract reduces life quality as it increases the risk of falls and fractures, affects daily life, and causes depression and anxiety [2]. Cataract also poses a heavy economic burden and substantial challenges for health systems [3]. Up to 1.2 million Australians aged 65 and above were affected by cataract in 2010 (https://aci.health.nsw.gov.au/ie/projects/falls-in-older-people-with-cataract), leading to an estimated total of direct and indirect costs of more than AUD 14·6 billion that year [4].

Cataract surgery is the most effective intervention to eliminate cataract-related visual impairment and blindness. Postoperative patients usually benefit from significantly improved visual function and quality of life [5]. In 2014, the cataract surgical rate in Australia reached around 8,000 per million population; it is estimated that over half a million people in Australia will have had cataract surgery by 2021 [6].

Despite extensive population-based studies investigating the individual risk factors for cataract surgery, the geographic disparity in the distribution of the surgery in Australia remains rarely elucidated [7–10]. Compared with individual-level studies, region-level studies are important as they can shed light on the incidence of cataract surgery (ICS) and its relationship to predictive factors from a regional perspective. Analyses of the temporal and geographic incidence rates will provide important information on the relative equity of ICS distribution, and its changes over time across different regions. This will enable health care stakeholders to identify the most critical areas for intervention and provide evidence for public policy-making to address geographic disparity [11].

New South Wales (NSW) is a state located in southeastern Australia, where 75% of the residents live in the Greater Metropolitan Region of Sydney [12]. It has been estimated that the proportion of its population aged over 65 years and older will grow from 14% in 2006 to 20% in 2030 (https://invest.nsw.gov.au/sector-opportunities/aged-care). The need for eye care services for age-related diseases is thus expected to grow across NSW.

Our study aimed to examine the temporal and spatial variations in ICS at a regional level using geographic information system (GIS) technology to determine if there are associations of the variations with socioeconomic status (SES) and/or private health insurance coverage in NSW.

## 2. Materials and Methods

### 2.1. Data Sources

The data used in this study were collected from the Sax Institute's “45 and Up Study,” a large-scale population-based prospective cohort study of individuals aged 45 and above in NSW, Australia (13). Participants were randomly sampled from the enrolment database of the Department of Human Services (DHS, formerly known as Medicare Australia). The overall response rate was 18%, and nearly 11% of the entire NSW population aged 45 years and older were included. Residents in regional and remote areas or those aged 80 and above were over-sampled. A total of 267,153 participants joined the study by completing a baseline questionnaire (distributed from January 2006 to December 2009) with a signed consent to link their information to the routine health databases. Details of the “45 and Up Study” are available in previous publications [13]. The “45 and Up Study” database was further linked to the Pharmaceutical Benefits Scheme (PBS) and the Medicare Benefits Schedule (MBS) databases. Thus, detailed information on medical procedures and medications prescribed could be tracked for each participant. The linkage of the “45 and Up Study” database to the MBS and PBS databases was done by the Sax Institute using a unique identifier provided to the DHS.

### 2.2. Ethical Approval

Ethical approval for the “45 and Up Study” was granted by the University of New South Wales Human Research Ethics Committee. Ethical approval for this specific study was granted by the Royal Victorian Eye and Ear Hospital Human Research Ethics Committee.

### 2.3. Geographic Measures

The Statistical Area 3 (SA3) level is a regional classification system for Australia's geographic areas that is based on data from the Australian Bureau of Statistics (ABS) and the Australian Standard Geographical Classification (ASGC). SA3 comprises a standardized set of numeric codes issued by the ABS to ensure the uniform identification of geographic entities. The delimitation of SA3s was based on the relative homogeneity of the population and function to identify regional characteristics. Individuals taking part in the study were assigned based on their residential postcode. In total, there were 91 SA3s in NSW, three of which (10702, 10803, and 12402) had fewer than 100 participants and were thus excluded from the final analysis. Digital boundary maps for 2011 that were used in the study were downloaded from the ABS (https://maps.abs.gov.au/index.html (Search: 2011 Statistical Area Level 3 and NSW)).

### 2.4. Identification of Private Cataract Surgery

Cataract surgeries performed in private hospitals from 2007 to 2016 were identified using the following MBS item codes: 42698, 42701, 42702, and 42716. We calculated the age- and sex-standardized cumulative ICS in each SA3 using a direct standardization technique based on the “45 and Up Study” population.

### 2.5. Inclusion and Exclusion Criteria

We included participants who had cataract surgery during the study period (from 2007 to 2016), and participants with the following conditions were excluded: (1) missing or invalid body mass index (BMI) or SA3 data; (2) holding a veteran's ID card; (3) a history of other ophthalmologic surgeries, including vitrectomy and cornea surgeries; (4) cataract-related eye diseases, including glaucoma and retinitis pigmentosa; (5) any other reported eye disease; and (6) participants from SA3s with fewer than 100 participants. After exclusions, a total of 234,201 residents were included for analysis in the study (Figure 1).

### 2.6. Influencing Factors

With the aim to explore the correlations between ICS and its influencing factors at a regional level, we analyzed regional economic covariates by two aspects: the SES indicated by the low index scores of socioeconomic disadvantages, the ratios of which were obtained from the participants' addresses linked to the indexes from the ABS, and the other being the extra private health insurance, the coverage of which was collected from the self-reported data derived from the baseline questionnaire. An SES index includes relative socioeconomic advantages and disadvantages, relative socioeconomic disadvantages, education and occupation, and economic resources. To determine the levels of regional SES with regard to cataract surgery, we chose the Socio-Economic Indexes for Areas (SEIFA) Index of Relative Socio-Economic Disadvantage (IRSD) (https://www.abs.gov.au/ausstats/abs@.nsf/DetailsPage/2033.0.55.0012011). With this measure, the lower the IRSD scores, the greater the disadvantages. For our analysis, we assigned each SA3 a score to represent its regional SES level, which was determined by the proportion of low-value IRSD (L-IRSD) scores of 1 or 2 in the region. Health insurance categories included private with extras, private with no extras, veteran's card (white or gold), health care concession card, and others. Extra private health insurance coverage was defined as the proportion of participants who held private health insurance with options for extra services.

### 2.7. Correlation Analysis

We assessed both nonspatial and spatial correlations. First, Spearman's correlation was used to determine if there was a nonspatial correlation between ICS and the influencing factors of cataract. Univariate Moran's I was applied to examine if there were any significant geographic variations in ICS, L-IRSD rate, and private health insurance coverage rate. Bivariate Moran's I was calculated to assess the colocation between ICS and each of the influencing factors. The measure of spatial correlation showed an indicator for spatial autocorrelation and evaluated whether the spatial pattern of a variable was clustered, dispersed, or random in the SA3s [14].

### 2.8. Local Indicators of Spatial Association

To visualize the clustering of variables and determine local clustering, a local indicator of spatial association (LISA) cluster map was created using a row-standardized spatial weight matrix based on rook contiguity. Spatial clusters visualizing the relationships between each of the influencing factors and ICS within the surrounding areas were produced using the bivariate LISA method [12]. To better illustrate changes in the geographic distribution of ICS over time in the LISA cluster map, we divided the study time frame into three periods: 2007–2009, 2010–2012, and 2013–2016. LISA analysis determined the boundaries between high (H) or low (L) levels of ICS and influencing factors in each SA3. For districts with significant correlations of ICS and insurance coverage rate, the LISA cluster maps illustrated significant correlations using the following labels: HH = high ICS/high insurance rate, LL = low ICS/low insurance rate, HL = high ICS/low insurance rate, and LH = low ICS/high insurance rate. These four groups were classified based on three norms. For instance, in a specific area to be classified as HL, bivariate local Moran's I was significantly different from zero and negative. In addition, the ICS of this specific area was significantly greater than the mean value of ICS, and the mean insurance coverage rate of the area adjacent to this specific area was lower than the mean value of the health insurance coverage rate [15].

### 2.9. Statistical Analysis

R Studio (version 1-1-463; *R* Studio, Inc., Boston, MA, USA) was used for data analyses. Ethnic variations in MBS claims were assessed using the chi-square test. Age- and gender-standardized ICS were calculated based on age and gender distributions from the 2011 census data. Range, mean, and standard deviation (SD) were evaluated to explore the statistical distributions of the outcomes and influencing variables. The spatial maps of outcomes and associated factors were plotted using ArcGIS 10.4 (ESRI, Redlands, CA, USA) and GeoDa 1.12 (Chicago, IL, USA).

## 3. Results

### 3.1. General Data of the Participants Involved in This Study

The present analysis involved a total of 232,201 people from 88 SA3s. The average number of participants per SA3 was 2,661 (95%CI, 508–6,925). The mean age of all participants was 62.4 (95%CI, 58.9–65.4), with 54% of participants being female and 75% being married. The average ICS occurrence between 2007 and 2016 was 8.85 percent (95%CI, 5.33–15.6). The mean proportion of individuals with L-IRSD was 20.5% (95%CI, 0.26–61.3) over the 88 SA3s, with 43.9% (95%CI, 20.8–74.1; Table 1) obtaining extra private health insurance coverage. The L-IRSD rate was found to be negatively correlated with ICS (*r* =  −0.25, *P* = 0.02, Spearman's correlation), suggesting socioeconomic conditions positively affect the cataract surgery service, while the number of people with additional private health insurance coverage was found to be positively associated with ICS (*r* = 0.25, *P* = 0.02, Spearman's correlation). The rate of L-IRSD was statistically inversely related to private insurance (*r* = −0.91; *P* < 0.001; Spearman's correlation; Table 1).

### 3.2. Variation of ICS by Geography

The geographical distribution of the ICS over a ten-year span is depicted in Table 1 and Figure 2. ICS showed a spatial distribution pattern that was significantly uneven despite the fact that there were few clusters (univariate Moran's I = 0.45, *P* = 0.001). At the SA3 level, all regions with a high ICS (sixth-quantile, brown shading) were located along the coast (Figure 2(a)). Based on Lisa analysis, six SA3s with a strong ICS (red shading) were identified in and around Newcastle, while 13 SA3s with a low ICS (blue shading) were identified in the suburbs of Sydney, Lachlan Valley (10302), and Dubbo (10503; Figure 2(b)).

### 3.3. Temporal Variation in ICS

Between 2007 and 2009, the coastal regions of NSW had the highest ICS rate. An HH clustering was detected in Newcastle and Lake Macquarie (11101, 11102, and 11103; Figure 3), and five LL SA3s were discovered in NSW's inland regions (11003, 11004, 10503, 10302, and 11301). From 2010 to 2012, ICS increased in Lower Murray, Upper Murray, Albury, and Wagga Wagga (10902, 10903, and 11303) but stayed unchanged in the state's south-west (10902, 10903, and 11303) (Figure 3(b)). On the LISA cluster map for 2013 to 2016, the HH clustering around Newcastle extended to include the Hunter Valley and the Mid North Coast (10601, 10602, 10603, and 10801, red shading) (Figure 3(c)). However, the strong tendency towards LL ICS clustering has waned over time, as shown by the absence of blue shading in the central regions of NSW, as a consequence of the rising ICS in Dubbo, Broken Hill, and Far West (10503 and 10502; Figure 3(c)) in the recent past. Over time, it has tended towards maintaining a balance around the whole state.

### 3.4. Colocation between ICS and Influencing Factors

The percentages of those with L-IRSD (univariate Moran's I = 0.45, *P* = 0.001) and others with extra private health insurance (univariate Moran's I = 0.58, *P* = 0.001) had a markedly disproportionate regional distribution. Additionally, important spatial correlations between ICS and the percentage of people with L-IRSD (bivariate Moran's I = −0.13, *P* = 0.009) and the percentage of people with additional private health insurance (bivariate Moran's I = 0.23, *P* = 0.001) were shown. According to our study, the frequency of L-IRSD and the proportion of additional private health insurance coverage had a significantly negative spatial relationship (bivariate Moran's I =−0.49, *P* = 0.001) (Table 1). The bivariate local Moran's I analysis, intuitively, showed a spatial association between ICS and its underlying causes. The bivariate LISA analysis of economic covariates revealed significant clustering areas of economic status among the 88 SA3s of the 10-year ICS: high ICS/low rate of L-IRSD high extra private health insurance coverage rate (same as high ICS/high economic status) in Sydney; high ICS/high rate of L-IRSD low extra private health insurance coverage rate (same as high ICS/low economic status) in Coffs Harbour (10402) and Port Macquarie (10804); and low ICS/low rate of L-IRSD low extra private health insurance coverage rate (same as low ICS/low economic status) in Armidale (11001), Moree-Narrabri (11003), and Richmond Valley (11201, 11202) (Figure 4). There was a colocation of association with high ICS/low economic status in Lower Murray and Griffith-Murrumbidgee, this was with the three quantiles of ICS (Figures 2(a) and 4(a)). It is distinct from the general situation due to the unknown additional driving factors in local ICS.

## 4. Discussion

In this Australian population, we found that ICS varied substantially across the state, with coastal regions covering most of the surgery cases, but the inequality decreased over time. In addition, there was a significant positive correlation between ICS and regional economic dynamics, especially in areas within and around Sydney.

A wide geographic variation in ICS across all SA3s was observed in the present analysis, with ICS gradually decreasing from the coastal regions to the northwest inland regions. Contrary to the remote SA3s in western and southern NSW, the SA3s in and surrounding Greater Sydney had greater population density. It is suggested that residents in these remote areas had less access to health care services than those in urban areas and therefore had not enjoyed the same benefits of increased awareness and improved diagnosis and treatment of cataract [16]. Furthermore, most hospitals within NSW are located in regions along the coast (https://www.myhospitals.gov.au/. 2019). These factors may partially explain the geographic imbalance in ICS observed in the current analysis. In addition, a clustered region of high ICS within and around the city of Newcastle was identified, which in turn suppressed the ICS in Hunter, the adjacent region. This implies that cataract patients living in Hunter might have driven a distance to undergo surgery in Newcastle. Furthermore, two LL regions, located in the Lachlan Valley and Dubbo SA3s, were identified in the middle of the state. To eliminate the geographic imbalance in ICS from the coastal region to the inland region, these two regions may warrant further policy attention in the future.

We also observed decreases in the inequality of ICS over time. Population migration might be closely associated with this development. Across NSW, around 90,000 residents moved into areas other than the metropolitan areas of Greater Sydney, Newcastle, and Wollongong [17]. A number of regions have undergone an average population growth of 10% per annum from 2006 to 2016, including Albury, Dubbo, Wagga Wagga, etc (https://www.nsw.gov.au/regional-nsw-today). In addition, ongoing high-level state government investment in health care and a focus on elective surgeries, such as cataract, and hip and knee surgeries, may have enabled certain patients to receive elective surgery faster than in the past (https://www.health.nsw.gov.au/news/Pages/20180827_00.aspx). This trend of migration and investment tended to eliminate low ICS in the middle of the state over time.

Our study also demonstrated a positive correlation between the economic status and ICS at the SA3 level, a negative correlation with L-IRSD score rates, and a positive correlation with extra private health insurance coverage rates, suggesting that basic health care services could be promoted through regional economic well-being. Although there was a low spatial coefficient between ICS and risk factors, geographic colocations and spatial concentrations/convergences revealed additional information in NSW in the bivariate local LISA maps. With the influence of marginality, there was an interesting strong correlation between ICS and economic status in the Greater Sydney area. Colocations of high ICS and high economic status (pink shading in Figure 4(a) and red shading in Figure 4(b)) indicated that ICS is substantially impacted by economic dynamics around Sydney.

This study has several strengths. To the best of our knowledge, it has the largest sample size for a spatial study designed to evaluate ICS at an SA3 level. Moreover, key data metrics, including predictive factors, have been defined and collected using standardized questionnaires. In addition to individual risk factors, the study utilized three important types of economic factors for cataract surgery—demographics, SES, and insurance—to respond to unity economic status. Finally, we applied bivariate Moran's I and bivariate LISA analysis techniques to evaluate the geographic variation for the two factors, and we can further intuitively grade.

It should be noted that there are several limitations. First, participants' statistical areas of residence were collected from the baseline questionnaire, and we could not account for participants who may have moved or passed away during the study period. Furthermore, these data relied on MBS item numbers coded, which only captured services paid for by DHS and be inferred from the procedure from private hospitals. Nevertheless, the combination of advantages, including shorter median waiting time and more flexible choices of surgeons and hospitals, has made private facilities the dominant setting for cataract surgeries in Australia [18]. According to a recent Australian report, over 70% of cataract patients now have surgery in a private facility [19]. Further studies are needed to confirm the current findings and ensure data from private hospitals remain applicable generally for patients throughout the state.

## 5. Conclusion

In conclusion, this study is one of the first large-scale studies to identify geographic disparities in ICS and its associations with economic status at SA3 levels. Findings from the study demonstrate that ICS varied substantially across regions of NSW, but inequality in surgery rates has decreased over time, with changes significantly correlated with the economic status. These results illustrate that further attention is needed to address geographic differences in cataract surgery in underserved areas, and future health policy must address these imbalances throughout the state.

## Figures and Tables

**Figure 1:** Study flow diagram. Inclusion and exclusion criteria of the study and methods of our statistical analysis.

**Figure 2:** 10-year incidence of cataract surgery among 88 SA3 areas. (a) The sixth-quantile map of the 10-year incidence of cataract surgery; (b) the LISA cluster map of the 10-year incidence of cataract surgery.

**Figure 3:** The incidence of cataract surgery in different time periods by among 88 SA3 areas. (a) The sixth-quantile map of cataract surgery incidence between 2006 and 2008; (b) the sixth-quartile map of cataract surgery incidence between 2009 and 2011; (c) the sixth-quartile map of cataract surgery incidence between 2012 and 2015; (A) the LISA cluster map of cataract surgery incidence between 2006 and 2008; (B) the LISA cluster map of cataract surgery incidence between 2009 and 2011; (C) the LISA cluster map of cataract surgery incidence between 2012 and 2015.

**Figure 4:** The bivariate local Moran's I analysis of 10-year incidence of cataract surgery by economic covariates among 88 SA3 areas. (a) The bivariate LISA cluster map of cataract surgery incidence by lowest SES and (b) the bivariate LISA cluster map of cataract surgery incidence by extras insurance.

**Table 1:** Regional characteristics of cataract surgery incidence and correlative factors in 88 SA3s in the “45 and Up Study”.

	Min	25th percentile	50th percentile	75th percentile	Max	Mean (SD)	Univariate		Bivariate		Spearman's correlation	*P* value
							Moran's I	*P* value	Moran's I	*P* value
Characteristics of the 88 SA3 regions
Number of participants	508	1416	2423	3589	6925	2661.38 (1459.9)
Mean age (y)	58.90	60.98	62.50	63.80	65.40	62.41 (1.64)
Female (%)	47.74	52.91	54.35	55.34	58.23	54.01 (2.00)
Married (%)	54.15	72.06	76.15	77.95	84.94	74.96 (5.41)
10-year ICS (%)	5.33	7.34	8.69	10.06	15.62	8.85 (2.10)	0.45	0.001
Economic covariates
Socioeconomic, low IRSD (%)	0.26	3.21	18.45	32.47	61.27	20.46 (17.47)	0.45	0.001	−0.13^#^	0.009	−0.25^#^	0.02
−0.49^	0.001	−0.91^	<0.001
Private insurance with extras (%)	20.80	35.18	42.76	52.09	74.05	43.88 (11.88)	0.58	0.001	0.23^#^	0.001	0.25^#^	0.02

Min = the smallest value in 88 SA3 regions; Max = the largest value in 88 SA3 regions. IC=incidence of cataract surgery; IRSD = Index of Relative Socio-Economic Disadvantage. ^*∗*^All with 5% confidence interval. ^#^Correlation with 10-year incidence of cataract surgery. ^ Correlation with private insurance with extras.

## Data Availability

The datasets used and analyzed during the current study are available from the corresponding author on reasonable request.
